# Functional Outcome and Inflammatory Response of Patients with Extra-Articular Distal Humeral Fractures following Implantation of Anatomically Precontoured Locking Compression Plates through a Posterior Approach

This article has been retracted.

**DOI:** 10.1155/2021/2426298

**Published:** 2021-07-28

**Authors:** Jingwei Wu, Limin Liu, Huaijian Hu, Zhihua Gao

**Affiliations:** Orthopedics Department, Xuanwu Hospital, Capital Medical University, Beijing, China

## Abstract

Distal humeral fractures are challenging injuries to surgically correct and account for up to 2% of all adult fractures. Surgical management of extra-articular distal humeral fractures is challenging considering surgical approach, implant selection, and position of the implant owing to the availability of different precontoured implants and plate configurations. Anatomically precontoured locking compression plates (APLCPs) allow the placement of angular stable screws right underneath the reduced joint surface fragments. To date, there is a lack of evidence supporting its superiority to conventional locking plate osteosynthesis (LPO) in treating extra-articular distal humeral fractures. The objective of the study is to evaluate the efficacy and safety of APLCPs in the treatment of extra-articular distal humeral fractures. A total of 100 patients diagnosed with humeral fractures and receiving treatments in our hospital between May 2018 and May 2020 fulfilled inclusion and exclusion criteria and were randomly assigned to LPO and APLCP groups according to the odd-even of the order of hospital admission, 50 cases per groups. Clinical endpoints were assessed including operation time; in-bed time; length of hospital stay; volume of intraoperative blood loss; VSA scores before and 24, 48, and 72 h after surgery; MEPS scores before and 3, 6, and 12 months after surgery; range of motion, flexion, and extension of the elbow; serum levels of CK, CRP, and IL-6; and incidence of complications after surgery. It was found that the APLCP group exhibited shortened operation time and in-bed time, decreased length of hospital stay, and reduced volume of intraoperative blood loss compared to the LPO group (all *P* < 0.001). The two groups had declined VSA scores concomitant with increased MEPS scores after surgery in a time-dependent manner (*P* < 0.001). Notably, the VSA scores in the APLCP group were all lower than those in the LPO group at indicated time points (24, 48, and 72 h) after surgery (*P* < 0.001). Besides, the MEPS scores in the APLCP group were all higher than those in the LPO group at indicated time points (3, 6, and 12 months) after surgery (*P* < 0.001). It was revealed that the patients receiving extra-articular distal humeral APLCP through posterior approaches exhibited greater ranges of motion, flexion, and extension of the elbow than those receiving LPO after surgery (*P* < 0.001). The patients receiving extra-articular distal humeral APLCP through posterior approaches exhibited lower serum levels of IL-6, CRP, and CK than those receiving LPO after surgery (IL-6: *P*=0.007, CRP: *P*=0.001, CK: *P*=0.001). The APLCP had a lower total incidence rate of complication than the LPO group (48.00% vs. 18.00%, *P*=0.003). In conclusion, these data support the notion that the implantation of anatomically precontoured APLCP through a posterior approach allows for improved functional outcomes and attenuated inflammatory response and prevents the incidence of postoperative complications compared to conventional LPO for internal fixation of extra-articular distal humeral fractures.

## 1. Introduction

The elbow joint is composed of distal humerus and proximal radius and ulna, including humeral ulnar joint, humeroradial joint, and proximal radioulnar joint, which are wrapped by the joint capsule. There are ligaments, synovial bursa, and muscles outside the capsule, involved in the support, protection, and movement of the joint [1]. The elbow joint was with a high incidence of fracture due to the particularity of anatomic location [2]. In 2005, Jeffrey Anglen has mentioned that about 7% of adults suffered from elbow fractures, including one-third suffering from distal humerus fractures [3]. The number of distal humerus fractures is increasing, probably associating with the growing elderly population over 65 years old [4]. However, young male patients with high-energy trauma were also involved in distal humerus fracture [5]. On the basis of the Orthopaedic Trauma Association's classification, distal humerus fractures are divided into three types, namely, extra-articular fracture, partial intra-articular fracture, and intra-articular fracture [6]. Extra-articular fracture was related to 16% of adult humeral fractures, 3% of all fractures as well [7], and it was hard to be treated because of its periarticular location, small distal fragments, osteoporotic characteristics in the elderly, and so on [8]. Intra-articular fracture is a complex injury, leading to a severe limit on the function of the elbow joint if it is not being well-treated [9]. Due to their crucial role in the ligament attachment and bony restraint for metacarpal translation of the lunar and ulnar bones, theoretically, these fractures contributed to the instability of the wrist joint and distal radioulnar joint [10]. Generally speaking, surgical treatment and nonsurgical treatment are the main potions for treatment of distal humerus fracture, and nonsurgical treatment would be a reasonable choice for distal humerus fracture patients with minimal or nondisplacement and surgical contraindications [4]. The majority of distal humerus fracture requires surgical intervention to restore the range of motion and function of the elbow joint. Although there is no conclusion about the best treatment for distal humerus fracture, two common surgical methods including an extramedullary fixation with an anatomical locking plate or intramedullary fixation with a nail were recommended [11]. In addition, the treatment of open reduction and internal fixation (ORIF) with plates and screws has been preferred in clinical for adults [9]. With the development of minimally invasive techniques, new implants have been developed and applied to fracture. Locking compression plate (LCP) is such a kind of new implant, which is completely changing the internal fixation of the plate [12]. Although various plate structures have been proposed for distal humerus fracture treatment, the optimal treatment for fixation of extra-articular distal humerus fracture remains a management dilemma. In this study, conventional LPO and APLCP fixations through posterior approaches were compared in patients with extra-articular distal humerus fractures, in order to confirm its efficacy; elbow joint function involving mobility, flexion, extension; and incidence of adverse reaction, which provided an optimum surgical protocol for extra-articular distal humerus fracture in adults.

## 2. Material and Method

### 2.1. Inclusion and Exclusion Criteria

All eligible patients should meet the following criteria: (1) the fracture of the humerus was diagnosed by X-ray film in lateral view of elbow functional position (elbow flexion 70–90°); (2) 24 ≤ age ≤ 69 years old; (3) fracture within three weeks; (4) body mass index ≤30 kg/m^2^; (5) complete clinical and follow-up data; (6) 12-month follow-up at least; and (7) informed consent signed by the patient or family members. Those patients were excluded if involved in the following criteria: (1) surgical contraindications; (2) moderate-severe osteoporosis; (3) history of humeral trauma; (4) serious dysfunction of heart, liver, kidney, lung, and so on; (5) mental disorder or cognitive impairment; (6) osteoarthritis and pathological fracture; (7) other elbow fractures; (8) another operative method adopted during surgery; and (9) follow-up not being processed.

### 2.2. Surgery Protocols

After admission, the relevant examination should be made to determine the fracture site and fracture type, and the corresponding treatment plan should be formulated according to the examination results. The patients in the LPO group were given a traditional locking plate, and the APLCP group was accepted locking compression plate through the posterior approach. All patients in the two groups of were treated with general anesthesia and tracheal intubation. The surgery was done by the same group of physicians.

The patients in the LPO group were maintained in a supine position with correct placement of affected limbs. The routine disinfection and isolation measure were carried out, and the air-pocket tourniquet was prepared for surgery. A surgical incision approach was performed along the posterior part of the affected area in patients. The muscle tissue was separated by blunt dissection and the periosteum was stripped to expose the fracture completely; finally, the small fracture fragments and surrounding necrotic soft tissue were removed. Humerus fracture was reset on the basis of the location and type of fracture. In brief, pulling the injured limbs downward and rotating the upper arm, after alignment of the intertubercular sulcus, the fracture discontinuity was inserted with a periosteal separator to reset by lever principle. After fracture reduction, one or two temporary Kirchner wires were used to fix humeral nodules. Lastly, under the guidance of a C-arm X-ray machine for examining reduction, the fracture was fixed with an appropriate locking plate. Subsequently, the tissue was sutured after the drainage tube was placed.

The patients in the APLCP group were placed in the lateral decubitus position and with shoulder abduction of 60° at the injured site and elbow flexion of 90°. The routine disinfection and isolation measure were conducted, and the air-pocket tourniquet was prepared before surgery. A 5 cm incision was made along the posterior part of the affected area in patients, and the skin and subcutaneous tissue were cut layer by layer to determine the position of the artery. In the process of separation, the radial nerve and peripheral artery should not be damaged, to ensure the adequate exposure of the fracture site in the operative field, and the small bone fracture fragments and surrounding necrotic soft tissue were removed. According to patients' fracture location and type, the reduction was done with the assistance of the C-arm X-ray, and butterfly bone was temporarily fixed with Kirschner wire. On the basis of the actual situation of the fracture, the locking compression plate with the appropriate size was selected and inserted into the radial nerve from the distal end of the incision. The temporary Kirschner wire was pulled out and screws were applied to fix the distal and proximal ends of the affected area. Finally, the incision was closed and the negative pressure drainage tube was indwelling to complete the surgery.

All patients have received antibiotics for 3–5 days, and the drainage tube was removed 2 days after surgery. Neurologic drugs were applied to patients with radial nerve injury. The affected limb was suspended for 4 weeks; the shoulder, elbow, wrist, and finger joint function exercise was performed at 3 d after surgery; and the exercise range can be gradually increased according to the patient's condition. The postoperative examination and rehabilitation exercise were used for the patients every month until recovery, and after recovery, load activity was started after examination in patients once every three months. The study was followed up for 12 months ending up in May 2021.

### 2.3. Clinical Endpoints

All patients' surgery time, intraoperative blood loss, postoperative hospital stay, postoperative bed time, and postoperative complications were recorded, including swelling of the fracture site, malunion, and wound infection. The way of serum sample was collected as follows: 3 ml of fasting venous blood was collected from each patient before and 1 d after surgery and was restored at a suitable temperature for coagulation; then, it was centrifuged for 10 minutes in a centrifuge with a 10 cm radius and with the speed of 2500 rpm/min. The levels of creatine kinase (CK), C-reactive protein (CRP), and interleukin-6 (IL-6) were measured by enzyme-linked immunosorbent assay (ELISA) using commercial kits (Beckman Coulter Co., Ltd., USA). The examination method of elbow joint motion was performed as the following criteria: the patient was kept in supine position with arm straightly placed along both sides of the trunk and palm clenched upward. The axis of the goniometer was located on the side of the elbow joint and passes through the epicondyle of the humerus, the fixed arm was parallel to the median line of the humerus, and the movable arm was parallel with the median line of the forearm, in order to record the activity of flexion, stretch, and elbow joint. Visual analogue scale (VAS) was adapted to evaluate pain intensity. Briefly, a 10 cm long scale with a sliding cursor was marked with 10 scales, and figures “0” and “10” were on both ends. The higher the figure was, the higher the pain level. Mayo Elbow Performance Score (MEPS) was used to evaluate the elbow joint function in terms of four aspects, involving pain, motion function, stability, and joint instability. The full score was 100, 90–100 was defined as excellent, 75–89 was thought to be good, 60–74 was considered as average, and score lower than 60 was bad.

### 2.4. Statistical Analysis

All data were processed by SPSS23.0 statistical software package, and the measurement data were calculated by mean ± standard deviation and were analyzed by *t*-test, and repeated ANOVA was used for comparisons at multiple time points. The counting data was described by pass rate or constituent ratio and examined by chi-square test. *P* < 0.05 was considered as a statistical difference.

## 3. Results

A total of 100 patients diagnosed with humeral fractures and receiving treatments in our hospital between May 2018 and May 2020 fulfilled inclusion and exclusion criteria and were randomly assigned to LPO and APLCP groups according to the odd-even of the order of hospital admission, 50 cases per groups. The study design is listed in Figure 1. The LPO group consisted of 27 males and 23 females, age ranging from 24 to 46 years and with an average age of 48.80 ± 5.10 years. There were 21 cases of right arm fractures and 29 cases of left arm fractures. According to the Association for Osteosynthesis/Association for the Study of Internal Fixation (AO/ASIF) classification, the LPO group contained 10 cases of A2 type, 8 cases of A3 type, 10 cases of B2 type, 7 cases of C1 type, 8 cases of C2 type, and 7 cases of C3 type; 14 cases of fall injury, 22 cases of traffic accident injury, 10 cases of crush injury, and 4 cases of others. The APLCP group comprised 30 males and 20 females, aged ranging from 26 to 68 years and with an average age of 48.50 ± 5.10 years. There were 22 cases of right arm fractures; 28 cases of left arm fractures; 9 cases of A2 type; 9 cases of A3 type; 11 cases of B2 type; 6 cases of C1 type; 9 cases of C2 type; and 6 cases of C3 type; 15 cases of fall injury; 21 cases of traffic accident injury; 11 cases of crush injury; and 3 cases of others. The LPO and APLCP groups could be comparable considering no significant difference in age, gender, fractured arms, AO/ASIF classification, and fractured reasons between the two groups (*P* > 0.05).

The operation time, in-bed time, length of hospital stay, and volume of intraoperative blood loss were (67.52 ± 2.51) min, (1.47 ± 1.56) d, (7.14 ± 0.53) d, and (249.84 ± 10.72) mL for the patients receiving extra-articular distal humeral APLCP through posterior approaches and (85.74 ± 2.43) min, (3.13 ± 1.23) d, (11.82 ± 0.61) d, and (315.52 ± 11.54) mL for the patients receiving LPO. It was found that the APLCP group exhibited shortened operation time and in-bed time, decreased length of hospital stay, and reduced volume of intraoperative blood loss compared to the LPO group (all *P* < 0.001), suggesting that patients with humeral fractures recovered faster when receiving extra-articular distal humeral APLCP through posterior approaches than LPO.

When assessing functional outcomes of patients with humeral fractures, the VSA scores before and 24, 48, and 72 h after extra-articular distal humeral APLCP through posterior approaches or LPO and the MEPS scores before and 3, 6, and 12 months after surgery were recorded. Before surgery, the two groups of patients had similar VSA and MEPS scores, showing no statistical difference (*P* > 0.05), while the two groups had declined VSA scores concomitant with increased MEPS scores after surgery in a time-dependent manner (*P* < 0.001, Tables 1 and 2). Notably, the VSA scores in the APLCP group were all lower than those in the LPO group at indicated time points (24, 48, and 72 h) after surgery (*P* < 0.001). Besides, the MEPS scores in the APLCP group were all higher than those in the LPO group at indicated time points (3, 6, and 12 months) after surgery (*P* < 0.001). As shown in Figures 2(a) and 2(b), the declines of VSA scores and the increases of MEPS scores were greater in the APLCP group than in the LPO group.

In addition to VSA and MEPS scores, the range of motion, flexion, and extension of the elbow were evaluated after extra-articular distal humeral APLCP through posterior approaches or LPO. The ranges of motion, flexion, and extension of the elbow were 109.52 ± 7.35°, 19.51 ± 4.42°, and 98.65 ± 11.24°, respectively, in the APLCP group, and 98.82 ± 6.46°, 15.35 ± 5.12°, and 81.21 ± 11.85°, respectively. It was revealed that the patients receiving extra-articular distal humeral APLCP through posterior approaches exhibited greater ranges of motion, flexion, and extension of the elbow than those receiving LPO after surgery (*P* < 0.001, Table 3).

Next, inflammation response was assessed by determining serum levels of IL-6, CRP, and CK in the patients after extra-articular distal humeral APLCP through posterior approaches or LPO. Before surgery, the serum levels of IL-6, CRP, and CK were (4.21 ± 0.84) pg/mL, (6.07 ± 0.92) mg/L, and (75.15 ± 13.15) IU/L in the APLCP group and (4.84 ± 0.72) pg/mL, (6.04 ± 01.01) mg/L, and (74.12 ± 13.17) IU/L in the LPO group. The two groups of patients had similar serum levels of IL-6, CRP, and CK, showing no statistical difference (*P* > 0.05). One day after surgery, the serum levels of IL-6, CRP, and CK were (45.58 ± 14.61) pg/mL, (21.17 ± 4.35) mg/L, and (181.79 ± 32.13) IU/L in the APLCP group and (73.03 ± 17.43) pg/mL, (38.14 ± 7.12) mg/L, and (273.52 ± 35.11) IU/L in the LPO group. The two groups had elevated serum levels of IL-6, CRP, and CK one day after surgery (*P* < 0.05). However, the patients receiving extra-articular distal humeral APLCP through posterior approaches exhibited lower serum levels of IL-6, CRP, and CK than those receiving LPO after surgery (IL-6: *P*=0.007, CRP: *P*=0.001, CK: *P*=0.001, Figures 3(a)–3(c)), indicating that extra-articular distal humeral APLCP through posterior approaches lead to attenuated inflammatory response, preventing patients from soft tissue injury.

The patients with humeral fractures suffered from several complications after surgery, including wound infection, radial nerve paralysis, malunion, and swelling of the fracture site. The total incidence rates of complications were 18.00% in the patients receiving extra-articular distal humeral APLCP through posterior approaches and 48.00% in the patients receiving LPO. The APLCP had a lower total incidence rate of complication than the LPO group (*P*=0.003, Table 4).

## 4. Discussion

Distal humerus fractures represent one of the most challenging orthopaedic injuries and pose a dilemma to surgeons. They are often multifragmented, occur in osteopenic bone, and have limited options for internal fixation due to complex anatomy. Conventional locking plate fixation of distal humerus fractures is often related to elbow stiffness, weakness, and pain. A painless, stable, and mobile elbow joint is desired after internal fixation as it allows the hand to conduct better activities of daily living. In this study, we compared functional outcome, inflammatory response, and the incidence of postoperative complications between patients with extra-articular distal humeral fractures following implantation of APLCPs through a posterior approach and LPO, in a bid to evaluate the efficacy and safety of APLCPs in treating extra-articular distal humeral fractures.

Plate fixation is commonly used to treat humerus fractures, while the ideal plate choice remains to be discussed. The mechanical stability in conventional plating depends on pressure to the surface of the bone [13]. The load transfer of axial forces from the bone to the plate and back to the bone is generated by the friction from the compression of the plate onto the bone surface. Screws are responsible for the compression between plate and bone, which engage bicortically in the bone [14]. The friction between bone and plate can be enhanced by contouring the plate to match the bone surface. The stability of fracture fixation in conventional plating can be further enhanced if the fracture ends are compressed. The mechanical environment that both fixation principles generate is the most important difference between conventional plating and locked plating. In contrast to absolute stability in conventional plating, locked plating requires relative stability with interfragmentary movement in the fracture gap which can easily exceed 2% of interfragmentary strain [15]. LCPs are cheaper and can be easily contoured, whereas APLCPs could provide better stability and therefore lower rates of mechanical failure. In the study reported by Prall et al., APLCPs prevent the subsidence of the reduced joint surface fragments more effectively and allow for improved patient outcomes when compared with conventional plates and screws [16]. In addition, Kumar et al. reported that LCP is a reliable option for achieving union in humeral diaphyseal nonunion, showing good functional outcomes in patients with higher physiological demands [17]. In our study, compared to LPO, shortened operation time and in-bed time, decreased length of hospital stay, reduced volume of intraoperative blood loss, declined VSA scores, increased MEPS scores, greater range of motion, flexion, and extension of the elbow were noted in patients receiving implantation of anatomically precontoured LCPs through posterior approaches. These data indicated that implantation of APLCPs through a posterior approach allows for improved functional outcomes of patients with extra-articular distal humeral fractures: (1) minimally invasive incision by APLCP benefiting the rehabilitation of patients; (2) reducing the soft tissue trauma to the patient; (3) maintaining the stability of the whole fracture site, keeping the normal blood supply of the body, and thus promoting bone healing; and (4) feasibility of early functional exercise after surgery to repair humeral fractures, concurring other results [18].

Distal humeral fractures are challenging to manage because the articular surfaces must be restored perfectly and following soft tissue injuries must be recognized and appropriately treated. Soft tissue injury is a risk factor to maintain the stability of the elbow joint after surgery [2]. Fracture-associated soft tissue injury triggers an inflammatory response in the host. Although the inflammatory response exerts beneficial effects at the site of the injury, such as wound healing and the elimination of exogenous microorganisms, an uncontrollable systemic inflammatory response may result in multiple organ failure [19]. We determined the serum levels of IL-6, CRP, and CK between patients 24 h after extra-articular distal humeral APLCP through posterior approaches and LPO. IL-6, CRP, and CK are three biology markers and their reductions were used to reflect less muscle damage caused by invasive orthopaedic surgery [20]. It was found that although the serum levels of IL-6, CRP, and CK were elevated 24 h after surgery, the patients receiving implantation of APLCPs through a posterior approach exhibited lower serum levels of IL-6, CRP, and CK compared to LPO, suggesting extra-articular distal humeral APLCP through posterior approaches leads to attenuated inflammatory response, preventing patients from soft tissue injury.

In summary, implantation of APLCPs through a posterior approach allows for improved functional outcomes, elicits a significantly reduced postoperative inflammatory response, causes less muscle damage, and prevents the incidence of postoperative complications compared to conventional LPO for internal fixation of extra-articular distal humeral fractures. Much attention should be paid during the implantation of APLCPs. Extensive dissection of the soft tissue should be avoided to protect the blood supply of the humeral head. When resetting the humeral head fracture block, the head shaft angle should be more than 120° to reduce the risk of fracture block displacement and internal fixation failure. Further study with a larger sample size and radiological data recording will have to validate the presented findings.

## Figures and Tables

**Figure 1:** The flow diagram of the study design.

**Figure 2:** The VSA scores of patients with humeral fractures before and 24, 48, and 72 h after extra-articular distal humeral APLCP through posterior approaches or LPO, and the MEPS scores before and 3, 6, and 12 months after surgery. ^∗^ indicates statistical difference when the LPO group was compared to the APLCP group at different time points.

**Figure 3:** The serum levels of CK, CRP, and IL-6 in the patients before and 24 h after extra-articular distal humeral APLCP through posterior approaches or LPO. ^∗^ indicates statistical difference when the LPO group was compared to the APLCP group 24 h after surgery.

**Table 1:** The VSA scores of patients with humeral fractures before and 24, 48, and 72 h after extra-articular distal humeral APLCP through posterior approaches or LPO.

Group	Before surgery	24 h after surgery	48 h after surgery	72 h after surgery
LPO (*n* = 50)	7.42 ± 1.92	4.25 ± 0.74^*∗*^	2.98 ± 0.27^*∗*^	2.54 ± 0.27^*∗*^
APLCP (*n* = 50)	7.32 ± 1.74	3.12 ± 0.76^*∗*^	2.34 ± 0.25^*∗*^	2.05 ± 0.26^*∗*^
*P*	0.785	<0.001	<0.001	<0.001

^∗^indicates statistical difference when compared with the former time point in the group.

**Table 2:** The MEPS scores of patients with humeral fractures before and 3, 6, and 12 months after extra-articular distal humeral APLCP through posterior approaches or LPO.

Group	Before surgery	3 months after surgery	6 months after surgery	12 months after surgery
LPO (*n* = 50)	57.43 ± 10.35	75.43 ± 4.52^*∗*^	84.56 ± 4.25^*∗*^	91.37 ± 3.58^*∗*^
APLCP (*n* = 50)	57.62 ± 10.24	81.78 ± 4.42^*∗*^	91.35 ± 4.98^*∗*^	96.58 ± 3.35^*∗*^
*P*	0.927	<0.001	<0.001	<0.001

^∗^indicates statistical difference when compared with the former time point in the group.

**Table 3:** The range of motion, flexion, and extension of the elbow after extra-articular distal humeral APLCP through posterior approaches or LPO.

Group	Range of motion (°)	Flexion (°)	Extension (°)
LPO (*n* = 50)	98.82 ± 6.46	15.35 ± 5.12	81.21 ± 11.85
APLCP (*n* = 50)	109.52 ± 7.35	19.51 ± 4.42	98.65 ± 11.24
*P*	<0.001	<0.001	<0.001

**Table 4:** The incidence rates of complications after extra-articular distal humeral APLCP through posterior approaches or LPO.

Group	Wound infection	Radial nerve paralysis	Malunion	Swelling of fracture site	Total rate
LPO (*n* = 50)	9 (18.00%)	5 (10.00%)	7 (14.00%)	3 (6.00%)	24 (48.00%)
APLCP (*n* = 50)	3 (6.00%)	2 (4.00%)	3 (6.00%)	1 (2.00%)	9 (18.00%)
*P*	—	—	—	—	=0.003

## Data Availability

The data used to support the findings of this study are included within the article.
